The article "Long non‐coding RNA Sox2 overlapping transcript (SOX2OT) promotes multiple myeloma progression via microRNA‐143‐3p/c‐MET axis" was retracted in 2023. Reasons: errors in the analysis; errors in the results or conclusions.

# Long non‐coding RNA Sox2 overlapping transcript (SOX2OT) promotes multiple myeloma progression via microRNA‐143‐3p/c‐MET axis

**DOI:** 10.1111/jcmm.15171

**Published:** 2020-03-21

**Authors:** Yu Tianhua, Li Dianqiu, Zhang Xuanhe, Zhang Zhe, Gao Dongmei

**Affiliations:** ^1^ Departments of Blood Transfusion China‐Japan Union Hospital of Jilin University Changchun China; ^2^ Ultrasonography Department China‐Japan Union Hospital of Jilin University Changchun China; ^3^ Shihezi University Shihezi China; ^4^ Department of Radiation Oncology China‐Japan Union Hospital of Jilin University Changchun China; ^5^ Department of Otorhinolaryngology The First Hospital of Jilin University Changchun China

**Keywords:** c‐MET, lncRNA, miR‐144‐3p, multiple myeloma, SOX2OT

## Abstract

Long non‐coding RNA Sox2 overlapping transcript (SOX2OT) was reported to be involved in progression of multiple cancers. However, the role and mechanism of SOX2OT in multiple myeloma (MM) has yet to be unravelled. In the present study, elevated SOX2OT levels are reported in MM cell lines and patient samples as compared to normal plasma cells (nPCs) and healthy donors, respectively. Knock‐down of SOX2OT led to a significant inhibition of cell proliferation, arrested cells at G0/G1 phase and induced cell apoptosis in MM samples in vitro, as well as slowed the growth of tumours in vivo. Additionally, our data indicated that SOX2OT functioned as a competing endogenous RNA (ceRNA) in MM cells that regulated miR‐144‐3p expression. Repression of miR‐144‐3p reversed the inhibition of MM development due to SOX2OT knock‐down. Our data also revealed that SOX2OT regulated the expression of the cellular‐mesenchymal to epithelial transition factor (*c‐MET*, a known target of miR‐143‐3p) by functioning as a sponge of miR‐144‐3p in MM samples. These data support that SOX2OT promotes MM progression through regulating the miR‐144‐3p/c‐MET axis, suggesting that SOX2OT might be as a potential therapeutic target for MM.

## 1 INTRODUCTION

Multiple myeloma (MM) is a disorder of the hematopoietic system involving the proliferation of cancerous plasma cells in the bone marrow.^1^ Despite recent advances in therapeutic interventions for MM and supportive strategies such as modulation of the immune system, inhibitors of the proteasome and stem cell therapy, the prognosis remains grim for MM patients due to the high incidence of relapse and resistance.^2^, ^3^ Therefore, understanding of the mechanisms associated with MM is needed to allow development of more effective treatment strategies.

Long non‐coding RNAs (lncRNAs) are more than 200 nucleotides in length that lack of protein‐coding capabilities.^4^ lncRNAs have been reported to play a vital role in various cellular processes including proliferation, death, apoptosis and invasion,^5^, ^6^ and reports have implicated lncRNA dysregulation in tumorigenesis, metastasis, disease diagnosis and prognosis of various cancers.^7^, ^8^ several studies report that aberrant lncRNAs are involved in the spread and advent of MM and may serve as useful biomarkers for therapy and prognosis.^9^, ^10^ Therefore, searching for novel targets from lncRNAs might be a promising therapeutic option for the treatment of MM.

SOX2 overlapping transcript (SOX2OT), located on chromosome 3q26.3, is a lncRNA transcribed in the same orientation as SOX2 that is embedded in an intron of the SOX2OT gene.^11^ SOX2OT has attracted growing attention due to its important role on the tumorigenesis of breast,^11^ gastric,^12^ ovary,^13^ lung,^14^ pancreatic ductal adenocarcinoma,^15^ colorectal cancer^16^ and so on,^17^, ^18^ suggesting that SOX2OT could serve as diagnosis marker and therapy target for various cancers. However, the precise role of this lncRNA in MM has yet to be determined.

Some lncRNAs were reported to serve as competing endogenous RNAs (ceRNAs) for sponging microRNAs (miRNAs) through their miRNAs response element (MREs), and sequester miRNAs away from their targets.^19^ The role of SOX2OT in the initiation and progression of oncogenesis via targeting several miRNAs, including miR‐363,^20^ miR‐194‐5p,^21^ miR‐132,^22^ miR‐122^23^ and miR‐211,^24^ has been reported. These studies suggested that SOX2OT could function as a ceRNA for sponging miRNAs. Through Starbase 2.0, we predicted that miR‐144‐3p could bind with SOX2OT. Growing evidence has suggested that miR‐144‐3p functioned as a tumour suppressor in various types of cancers by regulating cell proliferation, cell migration, migration apoptosis and angiogenesis.^25^, ^26^, ^27^, ^28^ A recent publication showed that miR‐144‐3p inhibited MM cell proliferation and induced cell apoptosis by targeting c‐MET (cellular‐mesenchymal to epithelial transition factor).^29^ However, the association with SOX2OT, miR‐143‐3p and c‐MET in MM remains unclear.

In this study, we explored the role and expression of SOX2OT in MM biology. We also examined the mechanism of regulation among SOX2OT, miR‐144‐3p and *c‐MET.* These results shed new light on a potential therapeutic intervention for MM.

## 2 MATERIALS AND METHODS

### 2.1 Patients

Thirty‐six MM patients (newly diagnosed IgG) were recruited from the China‐Japan Union Hospital of Jilin University during January 2014 to December 2017. All participants signed their informed consent. The mean age of MM patients was 57 (range: 38‐78 years), whereas the mean age of controls was 56.5 (range: 34‐75 years). Routine physical examinations were conducted. Samples from the bone marrow of 12 normal healthy donors (as control) and 36 MM patients were subjected to snap‐freezing in liquid nitrogen and stored at −80°C till further studies. All procedures were approved by the Institute Research Ethics Committee of Jilin University (Changchun, China).

### 2.2 Cell culture and assays

Four MM cell lines of human origin (ARP‐1, MM1S, U266 and NCI‐H929) and normal plasma cells (nPCs) were obtained from the American Type Culture Collection (ATCC, USA) and were maintained in RPMI‐1640 medium (KeyGEN Biotech) supplemented with 10% foetal bovine serum (FBS; Gibco), 100 U/mL penicillin and 100 mg/mL streptomycin in a 37°C humidified incubator with 5% CO_2_.

Short‐hairpin RNA (shRNA) targeting SOX2OT (sh‐SOX2OT) along with corresponding non‐targeting sequences (sh‐NC) was synthesized and inserted into the pGPU6/GFP/Neo vector (Gene‐Pharma, Shanghai, China). MM1S cells were transfected using Lipofectamine 2000 (Thermo Fisher Scientific) as per prescribed protocols. G418 (0.5 mg/mL; Sigma‐Aldrich) was used for selection of stably transfected cells. Mimics of miR‐144‐3p, the negative control mimics (miR‐NC) and the inhibitors of miR‐144‐3p (miR‐144‐3p in) with its negative control inhibitor (miR‐NC in) were obtained from Gene‐Pharma (Guangzhou, China). Transfection was done using the same method mentioned above. The efficiency of transfection was assessed by real‐time quantitative polymerase chain reaction (qRT‐PCR) 48 hours after transfection.

### 2.3 Real‐time quantitative PCR (qRT‐PCR)

Total RNA was extracted from cells and samples using with TRIzol reagent from Tiangen. Next, cDNA was synthesized using Qiagen's One Step PrimeScript cDNA kit (Hilden) as per the provided protocol. qPCR was performed using the SYBR Premix Ex Taq™ kit (TaKaRa) under the Applied Biosystems 7900 Sequence Detection (Applied Biosystems) as per prescribed instructions. TaqMan miRNA assay kits (Thermo Fisher Scientific) were used to assess levels of miR‐144‐3p. U6 was used as an internal control for miR‐144‐3p, and GAPDH was used for *SOX2OT* and *c‐MET* transcripts. The 2^−ΔΔCt^ method was applied to normalize levels of study mRNA as compared to the controls. The primers used in this study are listed in Table 1.

**TABLE 1:** Real‐time PCR primers used for mRNA or miRNA expression analysis

Target gene	Prime(5′‐3′)
U6	F‐ TCCGATCGTGAAGCGTTC R‐ GTGCAGGGTCCGAGGT
miR‐144‐3p	F‐ GCGCGCTACAGTATAGATGATG R‐ GCTGTCAACGATACGCTACG
SOX2OT	F‐ GCTCGTGG‐CTTAGGAGATTG R‐ CTGGCAAA‐GCATGAGGAACT
c‐MET	F‐ TGC ACA GTT GGT CCT GCC ATG A R‐ CAG CCA TAG GAC CGT ATT TCG G
GAPDH	F‐ AAGGTGAAGGTCGGAGTCAA R‐AATGAAGGGGTCATTGATGG

Abbreviations: F, forward; mRNA, messenger RNA; PCR, polymerase chain reaction; R, reverse.

### 2.4 Detection of cell proliferation capacity

MM1S cell proliferation was examined using a CCK‐8 kit (Cell counting kit‐8, Dojindo Molecular Technologies) according to manufacturer's protocols. Transfected cells were seeded into a 96‐well plate at 5.0 × 10^3^ per well and cultured for 24‐72 hours. This was followed by administration of 10 μL CCK‐8 reagent at culture incubation conditions discussed above for 4 hours. The absorbance at 450 nm was then recorded on a microplate reader (Bio‐Rad).

### 2.5 Flow cytometry assay to study cell apoptosis and cycle

To study cell cycle, transfected cells were harvested followed by an overnight suspension in ice‐cold 70% ethanol at 4°C. Cells were then washed twice using phosphate buffered saline (PBS) and incubated in 100 mg/mL propidium iodide (PI) from Beyotime (Beijing, China) along with RNase A (50 mg/mL, Beyotime) at 37°C for 30 minutes. The stages of the cell cycle were detected using the FACS Caliburflow cytometer (BD Biosciences) and the FlowJo7.6 analysis software tool.

The Annexin V‐FITC/PI Apoptosis Detection Kit (CWBIO) was used to assess apoptosis. To summarize, transfected cells were harvested and stained with fluorescein isothiocyanate (FITC)‐Annexin V and propidium iodide (PI) according to the instructions prescribed. The cell apoptosis ratio was determined using FACS Caliburflow cytometer (BD Biosciences) and the FlowJo7.6 analysis software tool (BD Biosciences).

### 2.6 Assay of luciferase reporter

Analysis with the Starbase2.0 (http://starbase.sysu.edu.cn/) predicted that SOX2OT would target miR‐144‐3p. The wild‐type sequence of SOX2OT including the potential site that targets miR‐144‐3p was synthesized and fused with the luciferase reporter vector pmirGLO from Promega and named: WT‐SOX2OT. The mutant sequence of SOX2OT was synthesized, then fused into the luciferase reporter vector pmirGLO and named: MT‐SOX2OT. Lipofectamine 2000 was utilized to cotransfect plasmids with WT‐SOX2OT or MT‐SOX2OT and miR‐144‐3p mimics or miR‐NC into MM1S cells for reporter activity assay. Luciferase activity 48 hours after transfection was assessed using the dual luciferase reporter assay system (Promega).

### 2.7 RNA immunoprecipitation assay

RNA immunoprecipitation (RIP) assay was performed using the Magna RIP RNA‐Binding Protein Immunoprecipitation Kit (Millipore) following prescribed protocols. Briefly, cells transfected with miR‐143‐3p mimic or miR‐NC were washed with pre‐cooled PBS and resuspended in lysis buffer. Cells were then incubated with RIP buffer containing argonaute2 (Ago2) antibody (or IgG antibody (both from Abcam) overnight. The enrichment of SOX2OT was measured from purified RNA using qRT‐PCR.

### 2.8 Tumour formation in mice models

A total of 20 male 4‐ to 6‐week‐old BALB/c‐nude mice were obtained from the Laboratory Animal Center of Jilin University at China and were housed individually under standard conditions in our laboratory. MM models were established by subcutaneous injection of MM1S cells which had been subjected to sh‐SOX2OT or sh‐NC transfection. Tumour volume was calculated every fifth day using the formula: Volume (*V*) = 0.5 × *a* × *b* ^2^, where *a* is the widest length and *b* represents perpendicular diameter. On the 30th day after injection, mice were killed and xenograft tumours were excised and weighed. A portion of these samples were fixed with 10% buffer formalin and stained for detecting Ki‐67 expression. The remaining tumour tissue samples underwent RNA extraction using RNA Trizol for further detecting SOX2OT, miR‐144‐3p and *c‐MET* mRNA expression by qRT‐PCR.

### 2.9 Immunohistochemistry assay

Expression of Ki‐67 was examined using immunohistochemistry (IHC) of mouse subcutaneous tumours as described previously.^30^ Ki‐67 antibody and secondary antibody were sourced from Santa Cruz Biotechnology Inc.

### 2.10 Statistical analyses

Data were presented as mean ± standard deviation (SD) of three independent experiments and processed using SPSS 19.0 software. Analysis among groups was performed using Student's *t* test or one‐way ANOVA. Correlation between SOX2OT and miR‐144‐3p/c‐MET was performed using Pearson's correlation analysis in the patient samples. *P* < .05 was considered significant.

## 3 RESULTS

### 3.1 Up‐regulation of SOX2OT in MM samples and cell lines

SOX2OT expression was measured in MM marrow samples (n = 36) as well as in control donor samples (n = 12) to characterize the role of SOX2OT in MM. qRT‐PCR showed that SOX2OT levels were higher in MM samples than in healthy samples (Figure 1A; *P* < .05). Additionally, the four human MM cell lines (ARP‐1, MM1S, U266, and NCI‐H929) had higher levels of SOX2OT than nPCs cells (Figure 1B). As MM1S cells had the highest SOX2OT expression, we selected MM1S cells for further experiments. These observations showed that SOX2OT expression is increased in patient samples and MM cell lines.

**FIGURE 1:** SOX2OT was up‐regulated in multiple myeloma (MM) samples and cell lines. A, Relative expression of SOX2OT in bone marrow from MM patients and healthy donors was determined by qRT‐PCR. GAPDH was used as an internal control. B, Relative expression of SOX2OT was examined four human MM cell lines (NCI‐H929, U266, MM1S and ARP‐1) and normal plasma cells (nPCs) by qRT‐PCR. GAPDH was used as an internal control. All data are presented as mean ± SD for at least three independent experiments, *P < .05, **P < .01

### 3.2 Knock‐down of SOX2OT suppressed proliferation of MM cells and induced apoptosis

MM1S cells were transfected with sh‐SOX2OT or sh‐NC to assess the role of SOX2OT in modulating MM cell cycle and apoptosis. As expected, knock‐down of SOX2OT caused a significant reduction in MM1S cells (Figure 2A). CCK‐8 assays showed that SOX2OT knock‐down obviously decreased cell viability of MM1S cells (Figure 2B; *P* < .05). Flow cytometry was performed to assess whether SOX2OT regulated the cell cycle or induced cell apoptosis. Analysis of the cell cycle revealed that MM cells arrested at G0/G1 phase when SOX2OT was knocked down, and the proportion of cells arrested at S phase was reduced (Figure 2C; *P* < .05). Assays for apoptosis revealed an increase in apoptotic MM cells due to silencing of SOX2OT (Figure 2C; *P* < .05). Hence, these observations show that SOT2OT knock‐down impaired proliferation and induced apoptosis in MM1S cells.

**FIGURE 2:** Knock‐down of SOX2OT suppressed MM cells proliferation and induced cell apoptosis. A, Relative expression of SOX2OT was examined in MM1S cells transfected with sh‐NC or sh‐SOX2OT by qRT‐PCR. GAPDH was used as an internal control. B‐D, Cell proliferation, cycle arrest and apoptosis were determined in MM1S cells transfected with sh‐NC or sh‐SOX2OT. All data are presented as mean ± SD for at least three independent experiments, *P < .05, **P < .01

### 3.3 SOX2OT acts as a molecular sponge for miR‐144‐3p in MM cells

We used bioinformatics tool (Starbase 2.0, http://starbase.sysu.edu.cn/) to predict miRNA that interacts with SOX2OT, revealing a potential miR‐144‐3p binding site in 3′UTR SOX2OT (Figure 3A). To confirm this, we performed a luciferase reporter assay in MM1S cells. We found that overexpression of miR‐144‐3p significantly reduced the luciferase activity of WT‐SOX2OT, not but that of MT‐SOX2OT (Figure 3B). An anti‐Ago2 RIP assay showed that endogenous SOX2OT was pulled down specifically in miR‐144‐3p overexpressed cells compared with miR‐NC group (Figure 3C). Moreover, overexpression of miR‐144‐3p significantly reduced SOX2OT expression (Figure 3D), and knock‐down of SOX2OT obviously increased miR‐144‐3p expression in MM1S cells (Figure 3E). Moreover, we determined miR‐144‐3p expression in MM patient bone marrow and cell lines. The results revealed that the expression of miR‐144‐3p was lower in bone marrows of MM patients and MM cell lines than that of health donors and nPCs, respectively (Figure 3F,G). Furthermore, the expression of SOX2OT and miR‐144‐3p was negatively correlated in patient bone marrow (Figure 3H). Taken together, these data suggest that SOX2OT functions as a molecular sponge for miR‐144‐3p in MM.

**FIGURE 3:** SOX2OT was a molecular sponge for miR‐144‐3p in MM cells. A, Schematic representation of the predicted binding sites between miR‐144‐3p and SOX2OT, and the mutagenesis design for the reporter assay. B, Luciferase activity was examined in MM1S cells after cotransfection with miR‐144‐3p mimic/miR‐NC mimic and reported plasmid WT‐SOX2OT or MT‐SOX2OT. C, The anti‐Ago2 RIP assay with miR‐144‐3p mimics revealed that both miR‐144‐3p and SOX2OT were enriched in Ago2 precipitate compared to control (IgG) in MM1S cells. GAPDH was used as an internal control. D, Relative expression of SOX2OT was measured in MM1S cells transfected with miR‐144‐3p mimic or miR‐NC by qRT‐PCR. GAPDH was used as an internal control. E, Relative expression of miR‐144‐3p was measured in MM1S cells transfected with sh‐SOX2OT or sh‐NC by qRT‐PCR. U6 was used as an internal control. F, Relative expression of miR‐144‐3p was measured in bone marrow from MM patients and healthy donors by qRT‐PCR. U6 was used as an internal control. G, Relative expression of miR‐144‐3p was examined four human MM cell lines (NCI‐H929, U266, MM1S and ARP‐1) and nPCs by qRT‐PCR. U6 was used as an internal control. H, Correlation between SOX2OT expression and miR‐144‐3p expression in bone marrow from MM patients was analysed by Pearson's correlation analysis. All data are presented as mean ± SD for at least three independent experiments, *P < .05, **P < .01

### 3.4 miR‐144‐3p inhibition alleviated SOX2OT knock‐down mediated inhibition of MM growth

To further explore whether SOX2OT exerts biological functions through miR‐144‐3p, we used rescue experiments by inhibiting miR‐144‐3p expression in SOX2OT knock‐down cells (Figure 4A). CCK8 assay showed reduced MM1S cell proliferation due to knock‐down of SOX2OT, and this effect was to some degree reversed by a miR‐144‐3p inhibitor (Figure 4B). Flow cytometry assays demonstrated that SOX2OT silencing causes a G1/G0 arrest, as well as induction of apoptosis in MM1S cells, and these results were also partially reversed in miR‐144‐3p inhibitor transfected cells (Figure 4C,D).

**FIGURE 4:** miR‐144‐3p inhibitor reversed the inhibitory effect of SOX2OT knock‐down on MM progression. A, Relative expression of miR‐144‐3p was measured in MM1S cells transfected with sh‐NC, sh‐SOX2OT with (without) miR‐144‐3p inhibitor(miR‐144‐3p in) by qRT‐PCR. U6 was used as an internal control. B‐D, Cell proliferation, cycle arrest and apoptosis were determined in MM1S cells transfected with sh‐NC, sh‐SOX2OT with (without) miR‐144‐3p in. All data are presented as mean ± SD for at least three independent experiments, *P < .05, **P < .01

### 3.5 SOX2OT modulated expression of c‐MET via miR‐144‐3p regulation in MM cell lines

Cellular‐mesenchymal to epithelial transition factor *(c‐MET)*, a known oncogene that promotes cancer progression in various cancers, has been shown to be a direct target of miR‐144‐3p in MM.^26^ Thus, we investigated whether SOX2OT regulated c‐MET expression in MM cells depended on miR‐144‐3p. We found that SOX2OT knock‐down caused a significant reduction in *c‐MET* levels, which were partially restored by miR‐144‐3p inhibitor in MM1S cells (Figure 5A). We then analysed the correlations among the expression levels of SOX2OT, miR‐144‐3p and *c‐MET* in MM specimens. qRT‐PCR analysis revealed a higher level of *c‐MET* in MM samples than in controls (Figure 5B). Further, Pearson's correlation analysis revealed that *c‐MET* expression was positively correlated with SOX2OT expression (Figure 5C) and negatively correlated with miR‐144‐3p in bone marrow specimens from MM (Figure 5D). These results suggest that SOX2OT negatively regulates miR‐144‐3p, leading to increase c‐MET expression in MM cells.

**FIGURE 5:** SOX2OT modulated c‐MET expression by regulating miR‐144‐3p in MM cell lines. A, Relative expression of *c‐MET* mRNA was measured in MM1S cells transfected with sh‐NC, sh‐SOX2OT with (without) miR‐144‐3p in by qRT‐PCR. GAPDH was used as an internal control. B, Relative expression of *c‐MET* mRNA was measured in bone marrow from MM patients and healthy donors by qRT‐PCR. GAPDH was used as an internal control. C, Correlation between SOX2OT expression and *c‐MET* expression in bone marrow from MM patients was analysed by Pearson's correlation analysis. D, Correlation between miR‐144‐3p expression and *c‐MET* expression in bone marrow from MM patients was analysed by Pearson's correlation analysis. All data are presented as mean ± SD for at least three independent experiments, *P < .05, **P < .01

### 3.6 Knock‐down of SOX2OT caused in vivo tumour suppression

Nude mice were injected with sh‐SOX2OT or sh‐NC‐transfected MM1S cells to study the function of SOX2OT on in vivo tumour growth. Xenograft tumour growth was examined every five days after inoculation. We found notably slower growth of tumours in the sh‐SOX2OT group as compared to the sh‐NC groups (Figure 6A, *P* < .05). At 30th day post‐injection, mice were killed and the tumours were excised and weighed. The results showed a notable decrease in tumour weight and size in the sh‐SOX2OT group as compared to the sh‐NC group (Figure 6B,C). Further, IHC revealed a decrease in the number of cells positive for Ki‐67 in the sh‐SOX2OT group compared to the sh‐NC group (Figure 6D). Moreover, qRT‐PCR examined the relative levels of SOX2OT, miR‐144‐3p and *c‐MET* expression in these xenografts tumour. The sh‐SOX2OT group showed a clear reduction in SOX2OT and *c‐MET* expression along with an elevation of miR‐144‐3p expression as compared to the sh‐NC group (Figure 6E). These data imply that SOX2OT knock‐down inhibits the growth of MM tumours in vivo.

**FIGURE 6:** Knock‐down of SOX2OT suppressed tumour growth in vivo. A, The tumour volume was measured every 5 d until mice killed. B, The tumour image. C, The tumours weight was measured. D, The Ki‐67 expression was determined in xenograft tumour by IHC. E, Relative expression of SOX2OT, miR‐144‐3p and *c‐MET* mRNA was measured in xenograft tumour tissues by qRT‐PCR. All data are presented as mean ± SD for at least three independent experiments, *P < .05, **P < .01

## 4 DISCUSSION

The involvement of lncRNAs either as oncogenes or as tumour suppressors in the initiation and progression of MM has been pinpointed by a growing amount of research.^9^, ^10^ For example, MEG3 serves as a tumour suppressor in MM to sponge miR‐181a and in turn regulate HOXA11, thus serving as a ceRNA.^31^ The growth of MM is supported by FEZF1‐AS1 via regulation of the miR‐610/Akt3 pathway.^32^ Another study showed that the PTEN/PI3K/AKT pathway is activated by targeting KLF10 through miR‐410 accumulation as induced by a loss of lncRNA OIP5‐AS1 ultimately leading to promotion cell proliferation and inhibition of cell apoptosis.^33^ Promotion MM cell proliferation and reduction in apoptosis was caused by Metastasis‐associated lung adenocarcinoma transcript 1 (MALAT1).^34^ The current study showed an up‐regulation of SOX2OT in MM samples as compared to controls. Knock‐down of SOX2OT reduced MM cell proliferation and induced cell apoptosis in vitro, along with an impairment of tumour growth in vivo. Further examination indicated that SOX2OT directly targeted miR‐144‐3p, which regulated c‐MET expression in MM cells. These observations support the potential role of SOX2OT as a therapeutic intervention in MM.

Numerous prior studies have implicated the up‐regulation of SOX2OT, a well‐known oncogenic lncRNA, in regulating cell proliferation, cycle arrest, apoptosis, migration, invasion and metastasis in multiple types of cancers.^12^, ^13^, ^14^, ^15^, ^16^, ^17^ However, the exact role and mechanism of this molecule has yet to be characterized in MM. This study showed an up‐regulation of SOX2OT in MM tumour specimens as well as cell lines as compared to their respective controls. Additionally, knock‐down of SOX2OT could suppress the growth of MM both in vitro and in vivo*,* as evaluated by CCK‐8 assay and by establishing xenograft tumours in nude mice. Cell apoptosis assays showed that knock‐down of SOX2OT induced MM cell apoptosis. This suggests that SOX2OT serves as an oncogene in MM progression.

We then investigated the miRNAs targeted by SOX2OT to assess its mechanism of action. Bioinformatics analysis showed a potential site for miR‐144‐3p to bind to SOX2OT, and further examination using luciferase and RIP assays supported SOX2OT as a direct target of miR‐144‐3p in MM cells. Our study has shown that the level of SOX2OT was reduced in the MM1S cells overexpressing miR‐144‐3p, whereas knock‐down of SOX2OT caused a notable increase in miR‐144‐3p. A negative correlation was observed between SOX2OT and miR‐144‐3p in MM bone marrow samples. Moreover, the growth inhibition due to knock‐down of SOX2OT was reversed by a miR‐144‐3p inhibitor in MM cells. These observations indicate that SOX2OT mediates its tumour‐promoting effects in MM cells through miR‐144‐3p. This study opens up new avenues of research into the pathway by which SOX2OT regulates miR‐144‐3p in tumorigenesis.

It was well known that lncRNAs, mRNAs and pseudogenes can communicate with each other by competing for MREs of miRNAs.^35^, ^36^, ^37^ As previously mentioned, the oncogenic role of SOX2OT was attributed to its ability to sponge out miR‐144‐3p in MM cells. c‐MET as a direct target of miR‐144‐3p has been previously confirmed in MM.^29^ c‐MET, a transmembrane receptor tyrosine kinase, was reported to be the receptor for hepatocyte growth factor (HGF).^38^ *c‐Met* has been identified to be up‐regulated and function as an oncogene in a variety of malignant including MM.^39^ Previous studies showed that inhibition of c‐MET by inhibitor or siRNA expression significantly inhibited MM progression by inhibiting cell proliferation and invasion.^40^, ^41^, ^42^ Thus, we further investigated whether SOX2OT could serve as a ceRNA to regulate *c‐MET* expression through competitive combination with miR‐144‐3p. Our results revealed that SOX2OT‐knock‐down in the MM1S cells significantly suppressed the levels of *c‐MET*, and this trend was rescued by miR‐144‐3p inhibitor. In addition, we found that *c‐MET* expression was up‐regulated in MM marrow samples and was positively correlated with SOX2OT. Therefore, the SOX2OT/miR‐144‐3p/c‐MET axis may function as an important player in MM progression.

In summary, the present study provides evidence that SOX2OT promotes MM progression through sponging miR‐144‐3p to regulate c‐MET (Figure 7). This provides novel insights into a critical role of SOX2OT as a miRNA sponge in MM and sheds new light on SOX2OT as a new a therapeutic target for MM.

**FIGURE 7:** Summary of the regulatory mechanism of SOX2OT in multiple myeloma

## CONFLICT OF INTEREST

The authors declare that they have no conflicts of interest.

## AUTHOR CONTRIBUTIONS

YT and LD designed the research directions and performed experimental contents. ZX contributed a lot to literature research and data analysis. ZZ and GD controlled the overall experimental direction.

## Data Availability

The data used to support the findings of this study are included within the article.
